# Traditional Chinese Medicine Ginseng Dingzhi Decoction Ameliorates Myocardial Fibrosis and High Glucose-Induced Cardiomyocyte Injury by Regulating Intestinal Flora and Mitochondrial Dysfunction

**DOI:** 10.1155/2022/9205908

**Published:** 2022-03-31

**Authors:** Junyan Wang, Peiwen Chen, Qiuyu Cao, Wei Wang, Xing Chang

**Affiliations:** ^1^School of Pharmaceutical Sciences, Guangzhou University of Chinese Medicine, Guangzhou 510006, China; ^2^The First Clinical Medical School, Guangzhou University of Chinese Medicine, Guangzhou 510405, China; ^3^Guang'anmen Hospital, Chinese Academy of Traditional Chinese Medicine, Beijing 100053, China

## Abstract

Myocardial fibrosis refers to the pathological changes of heart structure and morphology caused by various reasons of myocardial damage. It has become an important challenge in the later clinical treatment of acute myocardial infarction/ischemic cardiomyopathy or diabetes complicated with heart failure. Ginseng Dingzhi Decoction (GN), a Chinese herbal medicine, can reduce heart failure and protect cardiomyocytes. We infer that this may be related to the interaction with intestinal microbiota and mitochondrial homeostasis. The regulatory mechanism of GN on gut microbiota and mitochondria has not yet been elucidated. The intestinal microbiota was analyzed by the 16S rRNA gene; the fecal samples were sequenced and statistically analyzed to determine the changes of microbiota in the phenotype of heart failure rats. In addition, GN can regulate the microbial population that increases the proportion of short-chain fatty acids and anti-inflammatory bacteria and reduces the proportion of conditional pathogens to diabetic phenotype. The results suggest that GN may improve myocardial injury by regulating intestinal flora. Our data also show that stress-type heart failure caused by TAC (transverse aortic constriction) is accompanied by severe cardiac hypertrophy, reduced cardiac function, redox imbalance, and mitochondrial dysfunction. However, the use of GN intervention can significantly reduce heart failure and myocardial hypertrophy, improve heart function and improve myocardial damage, and maintain the mitochondrial homeostasis and redox of myocardial cells under high glucose stimulation. Interestingly, through in vitro experiments after TMBIM6 siRNA treatment, the improvement effect of GN on cell damage and the regulation of mitochondrial homeostasis were eliminated. TMBIM6 can indirectly regulate mitophagy and mitochondrial homeostasis to attenuate myocardial damage and confirms the regulatory effect of GN on mitophagy and mitochondrial homeostasis. We further intervened cardiomyocytes in high glucose through metformin (MET) and GN combination therapy. Research data show that MET and GN combination therapy can improve the level of mitophagy and protect cardiomyocytes. Our findings provide novel mechanistic insights for the treatment of diabetes combined with myocardial injury (myocardial fibrosis) and provide a pharmacological basis for the study of the combination of Chinese medicine and conventional diabetes treatment drugs.

## 1. Introduction

Diabetes combined with heart failure is one of the clinically common cardiovascular diseases that endanger the lives of patients [1, 2]. Although with the innovation of medical technology, most patients with diabetic cardiomyopathy can be admitted to the hospital for treatment in time and their condition can be stabilized, but there are still some patients with more severe myocardial hypertrophy, which later develops into severe heart failure [3, 4]. The further development of myocardial fibrosis (especially in the late stage of diabetic cardiomyopathy) can lead to severe decline or reduction of cardiac function, so myocardial fibrosis is also the pathological basis for the development and deterioration of diabetes complicated with heart failure [5]. Cardiomyocytes are terminally differentiated cells that cannot be regenerated. Once cardiomyocytes enter the process of apoptosis/necrotic apoptosis, they can only be replaced by scar tissue, which will cause structural and dysfunction of the heart, and eventually develop into heart failure [6, 7]. Different types of cardiomyopathy have different histological features, and myocardial fibrosis is common in many types of cardiomyopathy, often accompanied by the appearance of heart failure [8, 9].

Mitochondria are the main part of cardiac energy metabolism, and its dysfunction can lead to a variety of cardiovascular diseases [10, 11]. Mitochondrial homeostasis requires the coregulation of mitochondrial biogenesis, fusion, fission, and mitophagy to ensure the relative morphology, quantity, and quality of mitochondria stable to maintain the integrity of its structure and function [12, 13]. Mitochondrial homeostasis plays an important regulatory role in heart failure that occurs in the late stage of diabetic cardiomyopathy [14, 15]. This is mainly due to the fact that mitochondria can produce the most important energy substance in the heart-adenosine triphosphate (ATP), which is essential for maintaining the normal function of the heart [16]. Studies have shown that in a variety of myocardial injury diseases or in heart failure tissues that occur in the late stage of myocardial injury, the myocardial energy metabolism disorder caused by mitochondrial dysfunction can be observed [17].

Under the stimulation of inflammation or high glucose stress, the abnormal structure or function of mitochondria will not only lead to the disturbance of myocardial energy metabolism, but also produce a large number of reactive oxygen species (ROS) [18]. ROS can activate ryanodine receptor 2 and inhibit the activity of sarcoplasmic reticulum calcium transport ATPase, causing calcium overload of cardiomyocytes and decreased sensitivity of myofilaments to calcium [19]. Our previous studies have found that excess ROS will be accompanied by cells. Disorders of internal calcium homeostasis lead to increased levels of apoptosis and decreased levels of mitophagy [20]. Inhibition of mitophagy can lead to the failure of the damaged mitochondria of ischemia-reperfusion injury to be cleared in time, leading to mitochondrial homeostasis disorder, mitochondrial biosynthesis disorder, mitochondrial oxidative stress, mitochondrial membrane permeability transition pore (mPTP) opening, and accumulation of mitochondrial fragments, and eventually lead to mitochondrial apoptosis [21].

TMBIM protein, an evolutionarily conserved transmembrane Bax inhibitor, can mediate the process of cell death caused by Ca^2+^ release and calcium homeostasis disorder [22]. It can play an important role in regulating Bcl-2 protein in mitochondria, and TMBIM protein family can play a leading role in regulating both death receptor and endoplasmic reticulum calcium homeostasis [23]. TMBIM protein family widely exists in human/animal body or plant. TMBIM protein is a Bax sequence conservative inhibitor-1 (BI1 or TMBIM6), which can block Bax-induced cell death. TMBIM protein family (including TMBIM1/2/3/4/5/6) has an important feature that they can inhibit the excessive Ca^2+^ release in cells. TMBIM has a synergistic effect on the regulation of calcium balance [24]. In particular, TMBIM6, an important gene regulating endoplasmic reticulum, is an important intracellular calcium pool, so the calcium ion in endoplasmic reticulum must maintain a stable level to ensure the accuracy of calcium signal [25]. TMBIM6 can regulate the function of mitochondrion, which can control the Ca^2+^ overload in endoplasmic reticulum and the possibility of excessive Ca^2+^ entering mitochondria, so as to promote cell survival and make cells more resistant to the death stimulation mediated by calcium overload [26, 27]. Therefore, the specific mechanism of TMBIM6 in the process of cardiac fibrosis and cardiomyocyte injury mediated by mitophagy is very worthy of further explanation.

Ginseng internal flora Dingzhi Decoction (GN) is a myocardial protective drug extracted from the effective components of natural drugs such as ginseng, *Atractylodes macrocephala*, *Poria cocos*, yam, and xylooligosaccharide. Previous studies found that the effective components in the GN can play a regulatory role in improving the activity of cardiomyocytes and endothelial cells and maintain mitochondrial function and endoplasmic reticulum homeostasis through TMBIM6 [28]. Although the current research has preliminarily discussed the protective effects of mitophagy and mitochondrial dynamics on myocardial injury, the target drugs for mitophagy and diabetes mellitus complicated with heart failure are in short clinical. The aim of this study is to regulate the role of mitophagy in stress type heart failure and cardiac hypertrophy. Metformin hydrochloride (MET) is an important treatment for patients with diabetes and cardiovascular disease. For simple diet control and physical exercise treatment, invalid type 2 diabetes patients have very good treatment effect. Metformin can be combined with insulin to increase the hypoglycemic effect of insulin, reduce the amount of insulin, and prevent hypoglycemia. Metformin treatment of diabetes and myocardial injury is also found that MET can upregulate mitophagy, improve mitochondrial morphology and function, and maintain mitochondrial homeostasis and cell energy metabolism. Further studies also found that metformin can enhance autophagy and normalize mitochondrial function to reduce aging-related inflammation [29, 30].

For all that, the combined effect of metformin and Chinese herbal medicine is also very impressive, but its mechanism has not been verified by large-scale in vitro or in vivo experiments [31]. Therefore, this study verified the mechanism of GN improving myocardial injury and further explains the synergistic mechanism between GN and MET in order to provide a reference for diabetes mellitus complicated with myocardial injury.

## 2. Materials and Methods

### 2.1. PCR Amplification

The V3-V4 hypervariable regions of bacterial 16S rRNA gene were amplified with the primers 338F and 806R. For each sample, 10-digit barcode sequence was added to the 5′ end of the forward and reverse primers (provided by Expandbiotech, Life Science Park, Beijing, China). The PCR was carried out on a Mastercycler Gradient (Eppendorf, Germany) using 50 *μ*l reaction volumes, containing 5 *μ*l 10 × Ex Taq Buffer (Mg2 + plus), 4 *μ*l 12.5 mM dNTP Mix (each), 1.25 U Ex Taq DNA polymerase, 2 *μ*l template DNA, and 36.75 *μ*l ddH_2_O. Cycling parameters were 94°C for 2 min, followed by 30 cycles of 94°C for 30s, 57°C for 30s, and 72°C for 30s with a final extension at 72°C for 10 min. Three PCR products per sample were pooled to mitigate reaction-level PCR biases. The PCR products were purified using a QIAquick Gel Extraction Kit (QIAGEN, Germany), quantified using real-time PCR, and sequenced at Expandbiotech, Life Science Park, Beijing, China.

### 2.2. High-Throughput Sequencing

Deep sequencing was performed on MiSeq platform at Expandbiotech, Life Science Park (Beijing, China). After the run, image analysis, base calling, and error estimation were performed using Illumina Analysis Pipeline Version 2.6.

### 2.3. Sequencing Data Analyses

The raw data were first screened, and sequences were removed from consideration if they were shorter than 200 bp, had a low quality score (≤20), contained ambiguous bases, or did not exactly match to primer sequences and barcode tags. Qualified reads were separated using the sample-specific barcode sequences and trimmed with Illumina Analysis Pipeline Version 2.6. And then the dataset were analyzed using QIIME. The sequences were clustered into operational taxonomic units (OTUs) at a similarity level of 97%, to generate rarefaction curves and to calculate the richness and diversity indices.

### 2.4. Drugs and Concentration Selection

All drugs and natural active ingredient extracts were provided by Beijing Qianzhaoxinye Biotechnology and Co., Ltd. (Beijing, China) and passed the quality appraisal of Guangzhou University of Traditional Chinese Medicine. Ginseng internal flora Dingzhi Decoction (GN) mainly includes ginseng, *Atractylodes macrocephala*, *Poria cocos*, yam, and xylooligosaccharide.

### 2.5. Animal and Drug Intervention

All experiments were in accordance with the guidelines for laboratory animal care and use of the NIH and approved by the Guangzhou Committee for animal care and use of traditional Chinese medicine. Thirty male wild-type C57BL/6 J mice were obtained. Thirty C57 mice (8 week old) were randomly divided into sham operation group, TAC (transverse aortic constriction) operation group, and TAC + GN group. TAC + GN group (30 g/kg·d) was treated by gavage (15 days). The establishment of heart failure model in TAC group and TAC + GN group are referred to the previous work [32].

### 2.6. Grouping and Culturing of Cells

The cells were cultured at 37° C and 5% CO^2^. The medium was from Gibco (Grand Island, NY, USA) and contained 10% fetal bovine serum, 1% penicillin/streptomycin, and 0.1 mm norepinephrine and glutamine. Glucose is mainly provided by Sigma-Aldrich. Mouse cardiomyocytes were divided into control group, high glucose group, HG + GN group, and (4) HG + GN + si − TMBIM6 group. For small interfering RNA (siRNA) transfection, siRNAs were from Jikai Biology (Shanghai, China).

### 2.7. Cell Viability Assay

The activity of HL-1 cells was detected by MTT assay. Cells were inoculated into 12-well plates at a density of 50000 cells/well. The cell viability was detected by MTT method [28].

### 2.8. Flow Cytometry Detection

The apoptosis level of cardiomyocytes was detected by flow cytometry. The apoptosis detection kit was used for detection. Flow cytometer was used for automatic analysis of cells (Beckman, Brea, CA, USA) [33].

### 2.9. Detection of Oxidative Stress Markers

SOD and MDA kits were provided by Jiancheng Biotechnology Co., Ltd. (Nanjing, China). All test operations are carried out in accordance with the manufacturer's instructions. After collecting different groups of cells, ultrasonic was used for lysis reaction, then the cell lysate was centrifuged (3000°C and 20R/min), and then the supernatant was collected to detect the levels of SOD and MDA.

### 2.10. Laser Confocal and Immunofluorescence

After high glucose and drug pretreatment, the cells were washed with PBS and fixed with 4% paraformaldehyde. Then add 100 *μ*l first antibody and incubated at 4°C for 16 hours. The second antibody was then added. The fluorescence image was detected, and the average fluorescence intensity was analyzed by ImageJ software.

### 2.11. Q-PCR Detection

The total RNA of cardiomyocytes was extracted with TRIzol reagent and then reverse transcribed to synthesize cDNA under the catalysis of reverse transcriptase. Using cDNA as template, quantitative PCR was used for detection, the data was analyzed by 2^-△△CT^.

### 2.12. Western Blotting

The expressions of PINK (anti-PINK1 antibody (ab23707)), Parkin (anti-Parkin antibody (ab77924)), Drp1 (anti-DRP1 antibody (ab184247)), Mff (anti-Mff antibody (ab129075)), Fis1 (anti-FIS1 antibody (ab229969)), Bax (anti-Bax antibody (ab32503)), and *β*-actin (anti-beta-actin antibody (ab8226))were detected by western blotting. To be brief, cardiomyocytes were lysed using RIPA lysate (Beyotime, Shanghai, China). The supernatant was obtained by centrifugation (13000 g/30 min). Protein concentration was measured using BCA protein analysis kit. The same amount of protein was separated by SDS-PAGE and transferred to nitrocellulose membrane. After sealing with 5% skimmed milk powder, the membrane was incubated with primary antibody at 4°C overnight and then incubated with secondary antibody for 1 hour. Take photos and scan and quantify the optical density of the strip using ImageJ software.

### 2.13. Statistical Method

One-way ANOVA was used to compare multiple groups of data, and SNK-q was used to compare two groups of data. The significance criterion was **p** < 0.05.

## 3. Results

### 3.1. GN Improves Cardiac Function and Reduces Myocardial Fibrosis after TAC

Dysfunction of the heart often occurs in the process of diabetic cardiomyopathy or heart failure and is an important pathological mechanism. In order to observe the effect of GN on cardiac function and myocardial fibrosis injury after TAC, C57 mice underwent TAC operation and drug intervention. The results of echocardiography (Figures 1(a) and 1(b)) showed that cardiac function and ejection fraction gradually decreased after TAC in mice. Compared with the sham operation group, the cardiac function of TAC group deteriorated significantly, suggesting that TAC operation mice had a significant effect on cardiac function. However, the cardiac function and ejection fraction of mice after GN drug intervention were significantly improved (Figures 1(a) and 1(b)).

To verify the improvement effect of GN on myocardial injury, the myocardial tissues of mice in sham operation group, TAC, and GN drug intervention group were pathologically detected by Masson staining, H&E staining, and Sirius red staining. The experimental results showed that compared with the sham operation group, the myocardium of TAC group had serious myocardial injury and myocardial fibrosis/ventricular remodeling (Figures 1(c)–1(e)). However, the drug intervention of GN can improve myocardial injury and myocardial fibrosis/ventricular remodeling (Figures 1(c)–1(e)). Therefore, we infer that cardiac dysfunction after TAC may be related to myocardial injury and myocardial fibrosis, and GN can improve this pathological mechanism, protect myocardium, and inhibit the formation of myocardial fibrosis.

### 3.2. GN Can Inhibit the Synthesis of Collagenase in Damaged Myocardium and Improve Myocardial Hypertrophy

The increase of collagenase content or excessive deposition of collagen in cardiomyocytes is an important pathological mechanism leading to myocardial fibrosis or cardiomyocyte hypertrophy. We speculate that the improvement effect of GN on myocardial fibrosis may be related to its inhibition of excessive deposition of collagenase and synthesis of TGF-*β*. We first detected the expression levels of collagenase I and collagenase III in the myocardium of mice in each group by immunohistochemistry. We found that, compared with the sham operation group, the expression levels of collagenase I and collagenase III in the myocardium of TAC group increased significantly and the drug intervention of GN could inhibit the expression of collagenase I and collagenase III in the myocardium (Figures 2(a) and 2(b)). We further detected the transcription level of TGF-*α* and TGF-*β* by PCR. It was found that the transcription level of TGF-*α* and TGF-*β* in TAC group increased significantly, while the transcription level of TGF-*α* and TGF-*β* in GN group decreased significantly (Figures 2(c) and 2(d)). The results are consistent with those of immunohistochemistry, which suggests that GN can intervene the phenotypic transformation of cardiomyocytes and fibroblasts and play a certain regulatory role in the maintenance of cardiomyocyte function. We further detected cardiomyocyte hypertrophy by WGA immunofluorescence. It was found that cardiomyocytes in TAC group had significant hypertrophy and GN could reverse this phenomenon and maintain the stability of cardiomyocyte structure (Figures 2(e) and 2(f)).

### 3.3. GN Inhibits NLRP3-Mediated Inflammatory Response and Improves Cardiomyocyte Death of Mitochondrial Apoptotic Pathway

Inflammatory body (inflammasome) is an important component of inflammatory response. It is a complex composed of multiple proteins. It activates proinflammatory cytokines in a tolerant manner by caspase-1, including interleukin-1 *β* (IL-1 *β*), and induces inflammatory cell death. NLRP3 inflammatory bodies can have a significant impact on the regulation of mitochondrial homeostasis, and NLRP3 can stimulate the downstream common cellular signaling mechanism and interact with mitochondrial ROS. The blocking of mitophagy regulation pathway can also lead to the activation of NLRP3 inflammatory bodies. It mediates oxidative stress and inflammatory damage in myocardium and further mediates mitochondrial homeostasis dysregulation and cell death or apoptosis of mitochondrial pathway. We detected the expression levels of troponin and NLRP3 in mouse myocardium after TAC by immunofluorescence. We found that the expression of NLRP3 in mouse myocardium after TAC was significantly higher than that in sham operation group. However, GN could further inhibit the expression level of NLRP3 in myocardium after TAC (Figures 3(a) and 3(b)).

We further detected the myocardial tissue by TUNEL staining. We found that the positive proportion of myocardial tissue injury in TAC mice was large, and GN could reverse this phenomenon (Figures 3(c) and 3(g)). Q-PCR also found that the transcriptional level of caspase-3/-9/-12 in the myocardial tissue of heart failure mice increased to varying degrees, and GN could inhibit the transcriptional level of caspase-3/-9/-12 (Figures 3(d)–3(f)). The above results suggested that NLRP3-mediated inflammatory response and cardiomyocyte injury through mitochondrial apoptosis pathway may be the key mechanism of myocardial fibrosis injury and cardiac function in mice.

### 3.4. GN Regulates the Intestinal Microbial Community in Mice with Heart Failure

In order to determine the effect of GN on the composition of intestinal microbiota in different groups of mice, the feces of different groups of mice were detected by intestinal microbiota 16S technology. Diversity analysis showed that there were significant differences in the distribution of flora between the normal group and the model group, and there were differences in the diversity of intestinal microorganisms in each group (Figures 4(a)–4(h)) (*p* < 0.05). Moreover, the community composition structure of the four different groups of flora is also different, in which the difference between the normal group and the model group and between the high-dose group and the model group is very significant (Figures 4(a)–4(h)) (*p* < 0.05). On this basis, we further studied the differences of intestinal microbiota and different classification levels (Figures 5(a)–5(e)). We found that there were significant differences in flora classification between sham operation group and different dose groups (Figures 5(a)–5(e)) (*p* < 0.05).

To further study the effect of GN on intestinal flora in mice with heart failure caused by TAC, the ranges of different KEGG pathways and genes were determined. Through KEGG pathway detection, the experimental results show that the abundance of intestinal flora varied between groups (Figures 6(a)–6(e)) (*p* < 0.05). The experimental results confirmed that different doses of GN may further affect myocardial injury by regulating the abundance of intestinal flora with different functions. Studies have shown that some intestinal microbiota may affect colonization characteristics. During the treatment of myocardial injury or heart failure, the intestinal microbial community may change (Figures 4(a)–6(e)). We used 16S rRNA Gene Sequencing to identify key bacteria and possible changes in bacterial-related metabolic pathways. Compared with the control group, the low-dose group and high-dose group of GN improved the intestinal flora imbalance (Figures 4(a)–6(e)) (*p* < 0.05).

### 3.5. TMBIM6 Contributes to GN-Induced Protection against Cardiomyocyte Injury through Regulation of Redox Balance

Mitochondria are important organelles with double membrane structure in cells. Under normal physiological conditions, a small amount of electrons leak out from mitochondria in the process of electron transport capacity of respiratory chain, resulting in a small amount of ROS. A small amount of ROS, as a signal molecule, participates in the regulation of mitochondrial quality control, the activation of mitochondrial antioxidant system, and the regulation of cell proliferation crosstalk of differentiation, apoptosis, and other related signal pathways. The detection of caspase-3/-9/-12 suggests that myocardial injury may be closely related to mitochondrial apoptosis pathway. Therefore, through the transmission electron microscope detection of myocardial tissue of mice in different groups, it is found that mitochondria in myocardial tissue of mice after TAC appear expansion, deformation, and structural damage compared with sham operation group (Figure 7(a)). The structural changes of myocardial infarction area were observed by transmission electron microscope. It was found that cardiomyocyte dissolution or muscle fiber distortion was more serious, and mitochondrial structure was damaged and swollen in the TAC (Figure 7(a)). Interestingly, the intervention of GN can maintain the stability of mitochondrial structure and morphology (Figure 7(a)). In order to further verify the regulatory effect of GN on the activity and viability of cardiomyocytes, we stimulated cardiomyocytes with high glucose and detected the activity and apoptosis level of cardiomyocytes under different intervention conditions by MTT assay and flow cytometry. We found that different concentrations of GN had different effects on the improvement of cell activity; the cell activity of 200*μ*l group was the best (Figures 7(c) and 7(d)). Therefore, 200*μ*l medicated serum was used for intervention in the subsequent experiments. However, through the detection of cell viability and apoptosis level, it was found that the cell activity under high glucose stimulation decreased significantly, while the apoptosis level increased significantly, and GN could improve the cell activity under pressure stimulation and inhibit the apoptosis level (Figure 7(e)). Through the immunofluorescence detection of NLRP3, we found that the expression level of NLRP3 in cardiomyocytes will be further increased after high glucose stimulation. The experimental results suggest that the NLRP3-mediated inflammatory response under high glucose stimulation may be the main reason for the decline of cardiomyocyte apoptosis or activity (Figure 7(b)).

Interestingly, when high glucose stimulated cells were treated with GN pretreatment and siRNA-TMBIM6 at the same time, the cell activity decreased and the level of apoptosis increased significantly. We also detected the level of ROS production by flow cytometry. It was found that ROS was overaccumulated under the stimulation of high glucose. GN could inhibit the production of ROS, and the knockdown of tmbim6 could counteract the inhibition of GN on ROS (Figure 7(f)). This is consistent with the above results, which further suggests that the regulatory ability of GN on cell survival under stress stimulation is related to TMBIM6.

### 3.6. TMBIM6 Contributes to GN-Induced Protection against Cardiomyocyte Injury through Regulation of Mitochondrial Homeostasis

The mitochondria quality control and mitochondrial homeostasis are very important to maintain the basic viability of cardiomyocytes under pressure stimulation. Although the above experimental results preliminarily confirmed that apoptosis and excessive accumulation of ROS in mitochondrial pathway may be an important regulatory mechanism leading to cardiomyocyte death. However, whether the imbalance of redox balance mediated by mitochondrial energy metabolism and mitochondrial damage is involved in the protective mechanism of TMBIM6 has not been explained. Moreover, as the energy and metabolic center of cells, mitochondria have relatively independent quality control systems, including oxygen free radical scavenging system at the molecular level, fusion/fission mechanism at the organelle level, and mitophagy mechanism. The dysfunction of mitochondria and the imbalance of redox balance may be caused by each other. In order to verify the accuracy of the results of oxidative stress injury in cardiomyocytes, we detected the generation level of ROS in cardiomyocytes by ROS immunofluorescence. We found that the fluorescence intensity of ROS in cardiomyocytes under pressure stimulation was higher, while that in GN group was lower (Figures 8(a)–8(b)). This is consistent with the previous results of flow cytometry, and through the detection of SOD and MDA activity, it is found that SOD activity in high glucose group is inhibited and MDA is significantly increased, while GN intervention can improve SOD activity and inhibit MDA (Figures 8(c)–8(d)).

On this basis, we also detected the opening of mitochondrial membrane permeability transition pore (mPTP) and the level of mitochondrial energy metabolism by hippocampal detection system. The results suggest that under high glucose stimulation, mPTP will open abnormally, and the mitochondrial respiratory level and ATP production level have decreased significantly, while GN can inhibit the abnormal opening of mPTP and improve the mitochondrial respiration/ATP production (Figures 8(e)–8(g)).

It should be noted that the mechanism of GN effect on mitochondrial homeostasis in cardiomyocytes was reversed by TMBIM6 knockdown. siRNA-TMBIM6 treatment eliminated the regulatory effect of GN on redox balance mechanism and affected the protective effect of GN on mitochondrial energy metabolism and mitochondrial homeostasis in cardiomyocytes (Figures 8(a)–8(g)).

### 3.7. TMBIM6 Contributes to GN-Induced Protection against Cardiomyocyte Injury through Mitophagy and Mitochondrial Dynamics

Previous studies have explained the regulatory mechanism of mitochondrial homeostasis and mitochondrial oxidative stress on cardiomyocyte injury, but the regulatory mode of mitochondrial homeostasis and the therapeutic target of GN have not been further clarified. Under the normal metabolic state of cardiomyocytes, mitochondrial autophagy can clear mitochondria with abnormal or damaged structure and maintain the normal metabolic function of mitochondria. However, once the stress state exceeds the tolerance of mitochondria, it will lead to abnormal mitophagy, and the balance mechanism of mitochondrial fission and fusion will be broken, resulting in increased mitochondrial fragmentation and inhibition of mitochondrial autophagy. We first detected the protein expression level of mitophagy regulatory protein PINK/Parkin by western blot. We found that under the stimulation of high glucose, the protein expression level of PINK/Parkin decreased significantly, and GN could reverse this phenomenon (Figures 9(a)–9(g)). The results suggest that high glucose stimulation may reduce the level of mitophagy and GN may maintain mitochondrial homeostasis and mitochondrial function by improving mitophagy.

In order to further verify the role of mitochondrial dynamics in the regulation mechanism of GN maintaining mitochondrial homeostasis, we detected the protein expression levels of Drp1/Mff and Fis1. The results suggest that under the stimulation of high glucose, the protein expression levels of Drp1/Mff and Fis1 have increased significantly (Figures 9(a)–9(g)). The decrease of mitochondrial autophagy may be accompanied by the breaking of the balance mechanism between mitochondrial fusion and fission and the increase of mitochondrial fission level. However, the experimental results also found that the decrease of mitochondrial autophagy and the increase of mitochondrial fission level may mediate the increase of Bax (Figures 9(a)–9(g)). GN may block the mitochondrial apoptosis pathway related to Bax and caspase and protect cardiomyocytes by increasing mitophagy and inhibiting mitochondrial fission. Interestingly, knockdown of TMBIM6 eliminated the regulatory effect of GN on mitophagy/mito-fission (Figures 9(a)–9(g)) and blocking effect of GN on mitochondrial apoptosis pathway, which further verified the important role of TMBIM6 in the regulatory mechanism of GN protecting cardiomyocytes.

### 3.8. TMBIM6 Contributes to GN-Induced Protection against Cardiomyocyte Injury through Mitophagy and Mitochondrial Biosynthesis

Previous studies have explained the regulatory mechanism of mitochondrial homeostasis and mitochondrial dynamics in high glucose-induced cardiomyocyte injury. Once the stress state exceeds the tolerance of mitochondria, it will lead to abnormal mitophagy, resulting in increased mitochondrial fragmentation and inhibition of mitophagy. In order to detect the role of mitophagy in the regulatory mechanism of GN protecting cardiomyocytes, we first detected the transcription level of PINK/Parkin/ATG5/12 and PGC1*α* by Q-PCR. We found that under the stimulation of high glucose, the transcription level of ATG5/ATG12 and Pink/Parkin decreased significantly, and GN could reverse this phenomenon (Figures 10(a)–10(d)). The results suggest that high glucose stimulation may reduce the level of mitophagy, and GN may maintain mitochondrial homeostasis and mitochondrial function by improving mitophagy.

In order to further verify the role of mitochondrial biosynthesis in the regulation mechanism of GN maintaining mitochondrial homeostasis, we detected the transcription level of PGC1*α*. The results suggest that under the stimulation of high glucose, the transcription level of PGC1*α* have decreased significantly (Figure 10(e)). The decrease of mitophagy may be accompanied by the breaking of the mitochondrial biosynthesis. However, GN can increase the level of mitophagy and mitochondrial biosynthesis (Figures 10(a)–10(e)), and si-TMBIM6 could inhibit the regulation of GN on mitophagy and mitochondrial biosynthesis (Figures 10(a)–10(e)), which further verified the important role of TMBIM6 in the regulatory mechanism of GN protecting cardiomyocytes.

Through the immunofluorescence detection of NLRP3, the experimental results showed that the expression level of NLRP3 in cardiomyocytes stimulated by high glucose would be further increased, while GN could reduce the expression level of NLRP3 (Figure 10(f)). However, knockdown of TMBIM6 can counteract the therapeutic effect of GN and improve the expression level of NLRP3 (Figure 10(f)). Therefore, we infer that TMBIM6-dominated mitophagy (mediated by PINK/Parkin) may be an important way for GN to regulate the inflammatory response of cardiomyocytes stimulated by high glucose.

### 3.9. GN Can Enhance the Regulatory Effect of Metformin on High Glucose-Induced Cardiomyocyte Injury and Mitochondrial Homeostasis/Mitophagy Dysfunction

Metformin (MET) is a common hypoglycemic drug in clinic. It is mainly used in patients with type 2 diabetes mellitus who have poor diet control and high blood sugar, especially those with hyperlipidemia, obesity, and hyperinsulinemia. Current studies have shown that metformin can reduce the acute ischemic injury of a variety of organs such as the kidney, heart, and brain by regulating the transcription level of a variety of signal pathways and genes [29, 30]. Moreover, metformin has the characteristics of anti-inflammatory response and antioxidant stress and also has the effect of regulating mitophagy. This study verified that metformin could improve cardiomyocyte activity and redox balance stimulated by high glucose under different modes of GN/metformin coadministration and single administration. Both GN and MET can improve the activity of cardiomyocytes stimulated by high glucose and inhibit the overproduction of ROS. However, the combination of GN and MET can better regulate the improvement of cell activity and redox balance (Figures 11(a), 11(b), and 11(d)). In order to further verify the regulatory effects of GN and MET on mitophagy, we detected the transcriptional levels of PINK/Parkin, ATG5, and ATG12 by Q-PCR. The experimental results show that GN and MET can improve the transcriptional levels of PINK/Parkin, ATG5, and ATG12 to varying degrees. However, the combination of GN and MET can play a better regulatory role (Figures 11(c) and 11(e)–11(g)). This further confirmed the effectiveness of the combination of GN and MET, suggesting that metformin combined with GN can improve mitophagy level of cardiomyocytes, which provides a good reference for diabetic patients with diabetic myocardial injury.

## 4. Discussion

The results of this study show that the mitochondrial energy metabolism disorder mediated by mitophagy and mitochondrial fission dysfunction is closely related to the pathological mechanism of diabetic cardiomyopathy or myocardial fibrosis [34, 35]. Diabetes combined with heart failure is the end stage of many cardiovascular diseases such as diabetic cardiomyopathy or ischemic cardiomyopathy [36, 37]. The changes in the mechanical structure of the heart wall caused by the increase of long-term load pressure stimulation often develop into myocardial fibrosis and then gradually develop into heart failure [5, 38]. Under severe myocardial damage and metabolic dysfunction of myocardial cells, the ventricle will continue to change in size, shape, structure, and or abnormal local ventricular wall activity [39, 40]. Through in vitro and in vivo experiments and pathological/molecular biological detection methods, we verified the mechanism of GN improving myocardial injury and cardiomyocyte activity through TMBIM6-related mitophagy. We mainly verified three characteristics of the drug action of GN (GN combined with MET): first, GN can improve myocardial fibrosis and myocardial injury and is closely related to the regulation of mitochondrial structure and function; second, GN can improve mitophagy through TMBIM6, regulate the redox balance under high glucose stimulation, and improve the activity of cardiomyocytes under high glucose stimulation; third, the combined treatment of GN and MET can improve cardiomyocyte activity, which may be related to the inhibition of ROS outbreak and PINK/Parkin-mediated regulation of mitophagy.

Diabetic cardiomyopathy is described as a serious complication of late diabetes. Patients will develop heart failure and myocardial fibrosis without coronary artery disease, hypertension, and heart valve disease. The decline of cardiomyocyte function is an important mediating mechanism of heart failure. The decrease of cardiomyocyte function is partly caused by the abnormal structure or function of mitochondria. The pathogenesis of diabetic cardiomyopathy is complex, which is related to glucose and lipid metabolism disorders, insulin resistance, oxidative stress damage, and activation of NLRP3 and a variety of inflammatory pathways. Inflammatory pathways mediate cell and extracellular damage, cardiac remodeling, and relaxation and contraction dysfunction. Under the condition of diabetes, the energy metabolism function of myocardial cells is seriously affected. It leads to mitochondrial dysfunction and insulin resistance, endoplasmic reticulum stress (ERs), and cardiomyocyte apoptosis. The above factors usually affect each other and intensify, resulting in myocardial fibrosis, myocardial hypertrophy, myocardial ischemia, and abnormal cardiac diastolic and systolic functions, and finally develop into heart failure and myocardial fibrosis [41, 42]. The cytokines that induce heart remodeling and dysfunction can be derived from the heart, including cardiomyocytes, coronary microvascular endothelial cells, cardiac fibroblasts, and immune cells [43, 44].

In addition, our research results show that damaged myocardium can also release a large number of NLRP3 inflammasomes, which are the activation stimulating factors of NLRP3 inflammasomes. The activation of NLRP3 can accelerate cardiac remodeling and cardiac function disorders after myocardial infarction. Increased expression of NLRP3 protein and assembly of inflammasomes lead to caspase-1-mediated maturation and release of IL-1*β*, which triggers inflammation and pyrolysis. It plays a vital role in the process of myocardial fibrosis [45]. In myofibroblasts, NLRP3 inflammasome activation can cause the increase of activated IL-1*β*, which ultimately stimulates collagen synthesis, extracellular matrix protein expression, and myofibroblast differentiation, and participates in myocardial fibrosis and scar repair after myocardial infarction [46, 47]. There is also evidence that the sterile inflammatory response caused by tissue damage can be mediated by a multiprotein complex called NLRP3 inflammasome. Therefore, NLRP3 inflammasome may be the initial sensor of danger signals in myocardial ischemic injury [48]. It mediates the production of interleukin-1*β*, causes inflammation, and further aggravates inflammatory cell infiltration and cytokine expression [49, 50]. Interestingly, mitochondrial-derived reactive oxygen species (ROS) is a key signal that regulates the activation of NLRP3 inflammasomes. It is also a leading factor in the redox balance disorder.

In the current research results, our data show that in addition to the excessive production of ROS, there will also be the overexpression of oxidative stress markers and the decrease of antioxidant enzyme activity in the tissues or cells of myocardial fibrosis caused by pressure load [51]. At the same time, it will be accompanied by the imbalance of mitochondrial energy metabolism characterized by mitochondrial homeostasis; the changes of oxidative stress injury and mitochondrial homeostasis promote the process of myocardial injury and cardiomyocyte death [52]. The results preliminarily confirmed the regulatory mechanism of GN on redox balance and mitochondrial homeostasis. Increasing mitochondrial ROS and mitochondrial oxidative stress will affect or aggravate the damage of mitochondrial structure in the state of myocardial tissue or cell injury; this process may induce mitophagy or imbalance of mitochondrial fusion/fission mechanism [53]. If the damaged structure of mitochondria cannot be completely repaired, it will further affect mitochondrial energy metabolism and aggravate the excessive production of ROS [2], mediate the removal of mitochondria, fragmentation or damage useless mitochondria, and start the apoptosis of mitochondrial pathway [54, 55]. We found that GN can protect the ultrastructure of mitochondria by increasing the level of mitophagy, inhibiting mitochondrial fission and oxidative stress damage, maintaining the normal level of cell energy metabolism, and blocking mitochondrial cell apoptosis. At the same time, in vivo experiments confirmed that GN can well improve myocardial fibrosis and cardiac function and inhibit the activation of NLRP3 inflammasomes and the formation of myocardial collagen deposition. However, TMBIM6 plays an irreplaceable role in the myocardial protection mechanism and is an unimportant regulatory pathway for GN to treat diabetic cardiomyopathy or heart failure. TMBIM6 is an important mitochondrial function regulatory protein, which can maintain the normal function of cardiomyocytes by mediating mitophagy. It is expected to become an important intervention target for myocardial injury diseases or metabolic diseases in the future [56]. It has been found that TMBIM6/BI1 overexpression can inhibit the expression of myocardial XO, eliminate the excessive accumulation of ROS, block drp1-mediated mitochondrial fission, and protect myocardial injury and coronary microvascular injury caused by ischemia. This is consistent with our results. As a regulatory protein of mitochondrial homeostasis, TMBIM6 plays an indispensable role in the mechanism of GN maintaining mitochondrial function and protecting cardiomyocytes.

At present, the main drugs for the treatment of diabetes complicated with myocardial injury are hypoglycemic agents and insulin secreting agents. They all have some side effects and are prone to drug dependence. Therefore, the research and development of complementary and alternative drugs or synergistic drugs is an urgent problem to be solved. Natural drugs or Chinese herbal medicine can play the role of antioxidant, anti-inflammatory, antiapoptosis, immune regulation, and mitochondrial homeostasis regulation. And studies have found that the synergistic treatment of traditional Chinese medicine and Western medicine can play a better therapeutic effect.

Ginseng internal flora Dingzhi Decoction (GN), a traditional Chinese medicine prescription, Ginseng, Atractylodes macrocephala, Poria cocos, Yam and Xylooligosaccharides, etc. Currently, Ginseng internal flora Dingzhi Decoction as a protective drug for diabetes and myocardial damage. It can significantly reduce blood sugar and protect myocardium in both diabetic mice and myocardial injury mouse models. Under the intervention of the drug, the survival rate of mice is significantly improved. Ginseng internal flora Dingzhi Decoction also has the effects of intestinal flora and human intestinal microecosystem, which can promote the production of probiotics and inhibit the growth of pathogenic bacteria, thereby improving diabetes and obesity-related metabolic cardiomyopathy or metabolic syndrome. This study found that GN can further improve cardiac function and ejection fraction, effectively improve myocardial damage and myocardial fibrosis, and can also regulate myocardial redox balance and mitochondrial homeostasis. It is a therapeutic drug for diabetic cardiomyopathy with great potential. Previous studies have shown that puerarin (Pue), an effective ingredient in ginseng internal flora Dingzhi Decoction, can improve the mitochondrial respiratory function and energy metabolism of endothelial cells in an inflammatory state and increase cell activity. Quercetin (Que) in ginseng internal flora Dingzhi Decoction can inhibit H/R-induced cardiomyocyte oxidative stress damage through SIRT1/TMBIM6 and endoplasmic reticulum stress [28]. Studies have found that metformin can protect myocardial injury and cardiomyocyte injury after ischemia-reperfusion by inhibiting NLRP3 inflammatory bodies and activating AMPK [29].

In addition, it is also found that gut microbiota and its metabolites play an important regulatory role in cardiovascular disease. Intestinal microbiota imbalance has been recognized as an important pathological mechanism for the development of cardiovascular disease. Patients with cardiovascular disease are prone to intestinal barrier dysfunction due to reduced food intake and weakened intestinal mucosal regeneration. Studies have found that intestinal flora imbalance can be accompanied by oxidative stress injury, induce NLRP3 activation and lead to inflammatory response, and form vascular endothelial dysfunction and lipid/glucose metabolism disorder. Other related studies have found that the abnormality of intestinal flora is closely related to mitochondrial dysfunction. Intestinal microbiota may affect cell life and apoptosis by regulating mitochondrial function.

Gut microbiota has been shown to regulate key transcription factors, coactivators, and enzymes related to mitochondrial biogenesis and metabolism. In addition, microbiota metabolites seem to directly affect mitochondrial oxidative stress and the formation of mitochondrial autophagy lysosomes, thereby regulating the activation of inflammatory bodies and the production of inflammatory cytokines, which are the main factors of myocardial or cardiomyocyte metabolic disorder. Intestinal flora is the biological barrier of intestinal mucosa, and nutritional therapy is closely related to the maintenance of intestinal homeostasis. Enteral nutrition (EN) can better maintain the stability and balance of flora, while parenteral nutrition (PN) can significantly change the composition of flora and even aggravate the impairment of intestinal barrier function and bacterial translocation. Intestinal flora can affect mitochondrial function by regulating metabolites. Intestinal flora in different positions can decompose and release different metabolites, so as to realize the regulation of mitochondria. This study found that GN can regulate the distribution and abundance of intestinal flora in mice after TAC, and the abundance of intestinal flora in different groups is also different. Therefore, we infer that the regulation of intestinal flora may be one of the key therapeutic targets of GN. GN may regulate mitochondrial function and structure through intestinal flora and then affect mitochondrial energy metabolism and mitochondrial oxidative stress injury so as to protect cardiomyocytes.

Although this study conducted in vivo/in vitro experimental to explain the therapeutic mechanism of GN or GN combined with MET, there are still some limitations. First, we only validated the mechanism of GN on improving myocardial fibrosis through heart failure animal models and failed to verify the mechanism of GN in treating diabetic rats. This is very worthy of verification in the future. Second, the mechanism and effectiveness of GN and MET combination were verified only at in vitro experiments. No two drugs were used to treatment with myocardial injury or diabetic animal models. Third, because the pathological mechanism of diabetes complicated with heart failure is complex, it cannot be explained from the perspective of heart failure or high glucose-stimulated cardiomyocytes. Further studies should be carried out in order to provide more scientific and reasonable evidence.

In conclusion, our study shows that the effect mechanism of GN on improving myocardial injury and cell viability was verified both in vivo and in vitro through the regulation of intestinal flora or mitochondrial homeostasis. As shown in Figure 12, in the state of heart failure and stress-stimulated cardiomyocyte injury after TAC, NLRP3 can be activated and further affect mitochondrial homeostasis and inhibition of mitophagy, increase mitochondrial oxidative stress, and reduce mitochondrial energy metabolism; it is accompanied by the disorder of intestinal flora and finally leads to myocardial fibrosis/cardiomyocyte hypertrophy and aggravation of cardiomyocyte injury. GN can reverse this phenomenon, lead to improve cardiac function after TAC, regulate the distribution and abundance of intestinal flora, maintain mitochondrial homeostasis, improve mitochondrial function, improve mitophagy, inhibit oxidative stress, improve mitochondrial energy metabolism, protect cardiomyocytes, and reduce the level of myocardial fibrosis/hypertrophy. We further clarifies the protective mechanism of GN and MET (medication reconciliation) against metabolic cardiomyopathy or myocardial injury, which not only provides a reference for the future basic research of diabetes with myocardial injury and cardiovascular disease, but also provides guidance for the development of new targeted drugs.

## Figures and Tables

**Figure 1:** GN improves cardiac function and reduces myocardial fibrosis after TAC: (a) echocardiographic detection; (b) EF(%), FS(%), LVESV(*μ*l), LVEDV(*μ*l), E/A ratio, LVD-D(mm), LVD-S(mm), and myocardial fibrosis area (%); (c) hematoxylin-eosin staining; (d) Masson staining; (e) Sirius red staining. ∗*p* < 0.05.

**Figure 2:** GN can inhibit the synthesis of collagenase in damaged myocardium and improve myocardial hypertrophy. (a, b) The level of collagenase synthesis was detected by immunohistochemistry. (c, d) TGF-*β* 1 and TGF-*α* transcriptional level was detected by Q-PCR. (e, f) The hypertrophic and structure of cardiomyocytes were detected by WGA immunofluorescence. ∗*p* < 0.05.

**Figure 3:** GN inhibits NLRP3-mediated inflammatory response and improves cardiomyocyte death of mitochondrial apoptotic pathway: (a, b) immunofluorescence detection of NLRP3 in myocardial tissue, (c, g) TUNEL fluorescence detection of myocardial tissue, and (d–f) transcriptional level of caspase-3/-9/-12 in myocardial tissue. ∗*p* < 0.05.

**Figure 4:** GN changed the father of heart failure mice and changed the composition of intestinal microbiota community. (a–h) Differences in the abundance of specific intestinal microbial KO produced by TMAO. ∗*p* < 0.05.

**Figure 5:** GN changed the father of heart failure mice and changed the composition of intestinal microbiota community. (a–e) GN-induced functional changes of intestinal microbiota in mice with heart failure. ∗*p* < 0.05.

**Figure 6:** GN changed the father of heart failure mice and changed the composition of intestinal microbiota community. (a–e) Differential enrichment of specific gut microbial KOs for SCFAs production among four groups. ∗*p* < 0.05.

**Figure 7:** TMBIM6 contributes to GN-induced protection against cardiomyocyte injury through regulation of redox balance. (a) The morphology of mitochondria in myocardial tissue was detected by transmission electron microscope. (b) NLRP3 fluorescence intensity of cardiomyocytes was detected by immunofluorescence. (c, d) The activity of cardiomyocytes was detected by MTT assay. (e) The level of apoptosis was detected by flow cytometry. (f) The level of ROS production was detected by flow cytometry. ∗*p* < 0.05.

**Figure 8:** TMBIM6 contributes to GN-induced protection against cardiomyocyte injury through regulation of mitochondrial homeostasis: (a, b) ROS fluorescence intensity of cardiomyocytes was detected by immunofluorescence; (c) detection of antioxidant enzyme SOD activity; (d) detection of oxidative stress marker malondialdehyde (MDA); (e–g) detection of mitochondrial energy metabolism. ∗*p* < 0.05.

**Figure 9:** TMBIM6 contributes to GN-induced protection against cardiomyocyte injury through mitophagy and mitochondrial dynamics: (a) protein expression level of PINK/Parkin/Drp1/Mff/Fis1 and Bax was detected by western blot; (b) protein expression level of PINK; (c) protein expression level of Parkin; (d) protein expression level of Drp1; (e) protein expression level of Mff; (f) protein expression level of Fis1; (g) protein expression level of Bax; ∗*p* < 0.05.

**Figure 10:** TMBIM6 contributes to GN-induced protection against cardiomyocyte injury through mitophagy and mitochondrial biogenesis: (a) transcription level of PINK; (b) transcription level of Parkin; (c) transcription level of ATG5; (d) transcription level of ATG12; (e) transcription level of PGC1*α*; (f) NLRP3 fluorescence intensity of cardiomyocytes was detected by immunofluorescence. ∗*p* < 0.05.

**Figure 11:** GN can enhance the regulatory effect of metformin on high glucose-induced cardiomyocyte injury and mitochondrial homeostasis/mitophagy dysfunction: (a) CCK8 was used to detect cell activity; (b) MTT was used to detect cell activity; (c) transcription level of PINK; (d) immunofluorescence detection of ROS; (e) transcription level of Parkin; (f) transcription level of ATG5; (g) transcription level of ATG12. ∗*p* < 0.05.

**Figure 12:** In the state of heart failure and stress-stimulated cardiomyocyte injury after TAC, NLRP3 can be activated and further affect mitochondrial homeostasis and inhibition of mitophagy, increase mitochondrial oxidative stress, and reduce mitochondrial energy metabolism; it is accompanied by the disorder of intestinal flora and finally leads to myocardial fibrosis/cardiomyocyte hypertrophy and aggravation of cardiomyocyte injury. GN can lead to improve cardiac function, regulate the distribution and abundance of intestinal flora, maintain mitochondrial homeostasis, improve mitochondrial function, improve mitophagy, inhibit oxidative stress, and improve mitochondrial energy metabolism.

## Data Availability

The data used to support the findings of this study are available from the corresponding authors upon request.
